The article "Adverse Pregnancy Outcomes Associated with Endometriosis and Its Influencing Factors" was retracted in 2023. Reasons: signs of a paper mill; compromised peer review; unreliable results or conclusions.

# Adverse Pregnancy Outcomes Associated with Endometriosis and Its Influencing Factors

**DOI:** 10.1155/2023/7486220

**Published:** 2023-05-08

**Authors:** Li Xie, Yuanjie Qi, Hua Li, Li Chen

**Affiliations:** Department of Obstetrics and Gynecology, Fujian Maternity and Child Health Hospital, Affiliated Hospital of Fujian Medical University, Fuzhou, China

## Abstract

**Aim:**

To investigate the adverse pregnancy outcomes associated with endometriosis and its influencing factors.

**Methods:**

A total of 188 endometriosis patients who gave birth at our hospital between June 2018 and January 2021 were screened for eligibility and included in the research group, while a control group of 188 nonendometriosis women who delivered at our hospital during the same period were also included as healthy controls. Pregnancy outcomes were the key outcome measure, and the relationship between endometriosis and unfavorable pregnancy outcomes, as well as the influencing factors, were explored.

**Results:**

There was no significant difference in the risk of adverse pregnancy events such as miscarriage, ectopic pregnancy, termination of pregnancy, and fetal death between the two groups (*P* > 0.05). The differences in hypertensive disorder in pregnancy, gestational diabetes, placental abruption, fetal growth restriction, and luteal support between the two groups also failed to reach the statistical standard (*P* > 0.05). The two groups significantly differed in terms of cesarean delivery, preterm delivery, and placenta previa (1.92 (95% CI 1.33–2.85), 2.43 (95% CI 1.05–5.58), and 4.51 (95% CI 1.23–16.50)) (*P* < 0.05).

**Conclusion:**

Endometriosis is an influential factor in adverse pregnancy outcomes and results in a high risk of preterm delivery, placenta previa, and cesarean delivery in patients. Mutual interactions exist among adverse pregnancy outcomes and thus require appropriate management.

## 1. Introduction

Endometriosis [1] refers to the presence of endometrial tissue (glandular and mesenchymal) in the uterine cavity outside of the overlying endometrium and uterus, with recurrent bleeding and subsequent pain. It causes infertility and growth of nodules. Endometriosis has a high prevalence among women of childbearing age, and the lesion recedes after menopause. The disease is aggressive, recurrent, and sex hormone-dependent [2, 3]. Previous studies have shown that endometriosis increased the risk of several adverse pregnancy outcomes, such as preterm delivery, placenta previa, stillbirth, placental abruption, postpartum hemorrhage, and gestational diabetes [3, 4]. Moreover, Broi et al. [5] and Vercellini et al. [6] have reported an increased risk of hypertensive disorders during pregnancy. The size and depth of the peritoneal and ovarian lesions, the degree and extent of adhesion of the ovaries and fallopian tubes, and the magnitude of closure of the rectum and uterine pits are used for endometriosis classification. The most well-accepted notion of its pathophysiology is endometrial implantation [4].

The article "Adverse Pregnancy Outcomes Associated with Endometriosis and Its Influencing Factors" was retracted in 2023. Reasons: signs of a paper mill; compromised peer review; unreliable results or conclusions.

Pelvic pain is observed in 70–80% of the patients, including menstrual pain, chronic pelvic pain, painful intercourse, and anal cramps, infertility is found in 40%–50%, and 17–44% develop a pelvic mass (endometriotic cyst). It affects all pelvic tissues and organs, most notably the ovaries, uterine and rectal recesses, and uterosacral ligaments [5]. Periodic bleeding from the ectopic foci stimulates inflammatory reactions in the surrounding tissues, leading to adhesions in the pelvic cavity, which in severe cases compromises the peristalsis of the fallopian tubes or even leads to tubal obstruction. The preferred treatment option for endometriosis combined with infertility is laparoscopic surgery, which allows the diagnosis of the disease, removal of the lesion, and breakdown of adhesions, so as to improve the conception rate. However, the postoperative fertility rate remains unsatisfactory. In traditional Chinese medicine (TCM), the main pathogenesis of endometriosis is the stasis of blood blocking the ramus and the uterus. Endometriosis develops due to congenital deficiency of kidney essence, liver qi stagnation, and cold clotting of blood in the meridians. The patient's congenital deficiency of kidney essence, loss of both yin and yang, and inappropriate storage and drainage of the uterus result in stasis of the blood in the uterus. The patient's negative emotions, stagnant liver qi, and insufficient kidney yang lead to impaired warmth and aggravate the stasis of menstrual blood. Clinical treatments include surgery, medication, interventional therapy, herbal medicine, and adjuvant therapy (e.g., assisted reproductive technology treatment), so as to eliminate the lesions, reduce pain, ameliorate fertility, and avoid recurrence [6, 7].

Related research suggests a strong correlation between rectovaginal endometriosis and placenta previa [8]. Endometriosis may result in an increased risk of pregnancy complications [9], such as placenta previa, preterm delivery, hypertensive disorders of pregnancy, small gestational age, placental abruption, and postpartum hemorrhage. It is also considered to be associated with menstrual blood reflux [10]. Endometriosis is suggested to cause local immune and inflammatory responses via the production of cytokines, immune factors, and prostaglandins, resulting in a significant elevation of interleukin 1 and angiogenic factors in the peritoneal cavity, facilitating the adhesion of ectopic endometrial cells to the peritoneum, angiogenesis, and proliferation of ectopic endometrial lesions [11]. The significant elevation of cyclooxygenase 2, prostaglandin E and cytokines due to persistent immune, and inflammatory responses in the peritoneal cavity of patients with endometriosis may give rise to myometrial contraction and premature cervical maturation during pregnancy [12]. These aggravated inflammatory responses and growth factors on the uterine meconium and trophectoderm may also trigger adverse pregnancy outcomes.

The article "Adverse Pregnancy Outcomes Associated with Endometriosis and Its Influencing Factors" was retracted in 2023. Reasons: signs of a paper mill; compromised peer review; unreliable results or conclusions.

However, the contributory factors of endometriosis on perinatal outcomes are still poorly understood [13]. To this end, this study was undertaken to investigate the adverse pregnancy outcomes associated with endometriosis and its influencing factors, so as to provide relevant references for subsequent clinical treatment.

## 2. Materials and Methods

### 2.1. Participants

A total of 188 endometriosis patients who delivered at our hospital between June 2018 and January 2021 were screened for eligibility and included in the research group, whereas a control group of 188 nonendometriosis women who delivered at our hospital during the same period was included. The patients in the study group had endometriosis before pregnancy or ovarian endometriosis in early pregnancy, and they were treated accordingly.

The original sample size calculation estimated that 90 patients in each group would be needed to detect a 3-point difference between groups in a 2-sided significance test with a power of 0.8 and an alpha error level of 0.05.

Undersigned informed consent was obtained from the eligible patients prior to enrollment. The study protocol was approved by the Hospital Ethics Committee, and all processes complied with the Declaration of Helsinki ethical guidelines for clinical research.

### 2.2. Inclusion and Exclusion Criteria

#### 2.2.1. Inclusion Criteria

(1) Patients in the study group are those with pelvic endometriosis confirmed by histological examination [14]; (2) participants in the control group are those without confirmed endometriosis or any related ultrasound signs; (3) age ≤38 years, follicle-stimulating hormone <10 U/L, and endometrial thickness >8 mm on the day of progesterone conversion; (4) the patients were diagnosed with stage II EMT by laparoscopic surgery; and (5) prior to FET, vaginal ultrasound and hysteroscopy were performed without uterine malformations, endometrial polyps, and uterine adhesions.

#### 2.2.2. Exclusion Criteria

(1) Patients with combined malignancy; (2) with combined malignancy with multiple or multifetal pregnancies; (3) with autoimmune system diseases; (4) with adenomyosis; (5) with hydrosalpinx and without proximal tubal ligation or tubectomy; (6) with moderate to severe uterine adhesions and uterine malformations; (7) with comorbid medical conditions such as abnormal thyroid function, diabetes mellitus, and autoimmune system diseases; and (8) with hypercoagulated blood.

The article "Adverse Pregnancy Outcomes Associated with Endometriosis and Its Influencing Factors" was retracted in 2023. Reasons: signs of a paper mill; compromised peer review; unreliable results or conclusions.

### 2.3. Outcome Measures

Outcome measures include gestational age, mode of delivery, luteal support, and adverse pregnancy outcomes (preterm delivery, hypertensive disorders in pregnancy, gestational diabetes mellitus, placenta previa, placental abruption, and fetal growth restriction).

### 2.4. Definition

#### 2.4.1. Preterm Delivery

Delivery was performed before 37 weeks of gestation.

#### 2.4.2. Hypertensive Disorder in Pregnancy

It includes gestational hypertension and preeclampsia. Gestational hypertension refers to an increase in blood pressure of ≥140/90 mmHg after 20 weeks of gestation in a woman with previously normal blood pressure. Preeclampsia is gestational hypertension with proteinuria (≥300 mg/24 h).

#### 2.4.3. Gestational Diabetes

Gestational diabetes is diagnosed when any of the three values is met at 24–26 weeks of pregnancy, namely, fasting blood glucose ≥5.1 mmol/L, ≥10 mmol/L one hour after drinking sugar water, or ≥8.5 mmol/L two hours after drinking sugar water.

#### 2.4.4. Anterior Placenta

The placental tissue reaches or extends to the inside of the cervix [15].

#### 2.4.5. Placental Abruption

Bleeding at the meconium-placenta interface results in partial or complete detachment of the placenta before delivery.

#### 2.4.6. Fetal Growth Restriction

Fetal birth weight is lower than two standard deviations from the mean weight for the same gestational age or less than the 10th percentile of the normal weight for the same age.

### 2.5. Statistical Analysis

Logistic regression was used to analyze the adverse pregnancy outcomes and influencing factors associated with endometriosis, and SPSS 22.0 software was used to process the data and statistical analyses. The measurement data were expressed as (mean ± standard deviation) and analyzed by the independent sample *t*-test. Count data were expressed as number of cases (%) and analyzed by the chi-square test. *P* < 0.05 suggested that the difference was statistically significant.

## 3. Results

### 3.1. Patient Characteristics

There were 188 patients in the study group, aged 25–38 (30.96 ± 3.32) years, with a gravidity of 1–3 (1.56 ± 0.23). There were 25 cases with a BMI <18.5, 128 cases with a BMI of 18.5–23.9, and 35 cases with a BMI >24. There were 188 participants in the control group, aged 23–38 (30.23 ± 2.98) years, with a gravidity of 1–3 (1.41 ± 0.35). There were 26 cases with a BMI <18.5, 125 cases with a BMI of 18.5–23.9, and 37 cases with a BMI >24. The patient characteristics of the two groups were comparable (*P* > 0.05). (Table 1).

The article "Adverse Pregnancy Outcomes Associated with Endometriosis and Its Influencing Factors" was retracted in 2023. Reasons: signs of a paper mill; compromised peer review; unreliable results or conclusions.

### 3.2. Pregnancy Outcome

#### 3.2.1. Maternal Pregnancy Outcome

There was no statistically significant difference in the risk of miscarriage, ectopic pregnancy, pregnancy termination, or fetal mortality between the two groups (*P* > 0.05). (Table 2).

#### 3.2.2. Adverse Pregnancy Outcomes

The differences between the two groups in hypertensive disorder in pregnancy, gestational diabetes, placental abruption, fetal growth restriction, and luteal support did not meet the statistical standard (*P* > 0.05), but the differences in cesarean delivery, preterm delivery, and placenta previa were statistically significant (1.92 (95% CI 1.33–2.85), 2.43 (95% CI 1.05–5.58), and 4.51 (95% CI 1.23–16.50)) (*P* < 0.05). (Table 3).

## 4. Discussion

Endometriosis is the presence of the endometrial tissue (glandular and mesenchymal) in the uterine cavity outside the overlying endometrium and uterus [15]. The diagnosis of endometriosis requires the laparoscopic examination of visible pelvic lesions and biopsies of the lesions [16]. The increased use of human-assisted reproductive technologies has significantly boosted pregnancy success rates in patients with endometriosis, and there is also an escalating incidence of adverse pregnancy outcomes due to adverse reactions caused by endometriosis [17]. Endometriosis may lead to pregnancy failure or complications in late pregnancy. The local immune and inflammatory response to endometriosis significantly increases the levels of intraperitoneal IL-1*β* and angiogenic factors, which favor ectopic endometrial cell adhesion, proliferation, and angiogenesis. Thus, the local immunological and inflammatory response to endometriosis has a long-term impact on pregnancy and progesterone resistance, irregular uterine contractions, and thickening of the uterine junctional zone all threaten embryo implantation. The relationship between endometriosis and poor pregnancy outcomes, however, remains uncertain. Previous research has implicated endometriosis with the development of unfavorable pregnancy outcomes [18].

Previous studies suggest that chronic inflammation, uterine hormone-resistant endometrium, and the vascularized environment are associated with complications during pregnancy. In addition, abnormalities in the endometrium and the junctional zone at the molecular and functional levels lead to impaired endometrial growth, maturation and ecdysis, endometrial tolerance, defective spiral artery remodeling, and deep placental defects [19]. Preeclampsia is characterized by abnormal vascular remodeling, which is linked to a variety of pregnancy problems, including premature birth and fetal development limitation. As a result, it is theorized that placental anomalies are associated with an increased risk of placental problems and that endometriosis initiates a persistent pelvic inflammatory process. The increased number of prostaglandins and cytokines in endometriosis patients' peritoneal fluid increases myometrial contraction and cervical maturation, resulting in premature birth [22, 23]. In addition, alterations in the frequency and amplitude of uterine contractions in women with endometriosis cause dysfunction of the uterine tissues, which contributes to the increased risk of placenta previa. Due to extensive pelvic adhesions, placenta previa may also hinder placental migration from the intrauterine aperture. The higher incidence of placenta previa in endometriosis patients treated surgically before pregnancy is attributed to severe endometriosis or a high incidence of recurrence. The association between preconception surgery for endometriosis and the risk of placenta previa has been marginally explored [24, 25].

The article "Adverse Pregnancy Outcomes Associated with Endometriosis and Its Influencing Factors" was retracted in 2023. Reasons: signs of a paper mill; compromised peer review; unreliable results or conclusions.

Surgery is currently the main treatment modality for endometriosis-related infertility, and laparoscopic surgery can increase the pregnancy rate to 46.09%. Laparoscopic surgery is currently the gold standard for the diagnosis and treatment of endometriosis, with minimal gas trauma and short healing time, during which the ectopic foci visible to the naked eye can be removed and the mutual adhesions between tissues can be separated, so as to restore the anatomical structure of the pelvis. One of the causes of infertility in patients is the altered pelvic microenvironment, and intraoperative saline irrigation of the pelvis to improve its microenvironment is the major merit of laparoscopic surgery. However, laparoscopic surgery is insufficient for the removal of microscopic lesions and atypical ectopic lesions, so postoperative adjuvant medication is required. TCM classifies endometriosis as “infertility” and “menstrual disorders” according to its symptoms. According to the ancient medical books of TCM, if the pain occurs before menstruation, it is a factual pain and the pain will be relieved if the menstrual blood is discharged on time. If the pain occurs after menstruation and the pain persists after the discharge of menstrual blood, it is deficient pain. Diagnosis of the specific disease requires the clinical assessment of the patient's clinical symptoms.

The results of this study showed that there was no significant difference in the risk of events such as miscarriage, ectopic pregnancy, termination of pregnancy, and fetal death between the two groups, and the differences in hypertensive disorder in pregnancy, gestational diabetes, placental abruption, fetal growth restriction, and luteal support between the two groups also failed to meet the statistical standard (*P* > 0.05), while the incidence of cesarean delivery, preterm delivery, and placenta previa differed significantly between the two groups (1.92 (95% CI 1.33–2.85), 2.43 (95% CI 1.05–5.58), and 4.51 (95% CI 1.23–16.50)), which may be attributed to the imbalance of progesterone receptor subtype ratios in patients with endometriosis, causing progesterone resistance [24] and abnormal autoimmune response, inducing an increase in abdominal macrophages and the secretion of a large number of cytokines [25], such as prostaglandin F2*α*. Prostaglandin F2*α* levels are significantly elevated in the peritoneal fluid of patients with endometriosis relative to normal women, and prostaglandin F2*α* binds to the receptor and activates nucleic acid endonucleases that break DNA, leading to decreased blastocyst formation and quality. Multiple factors interact with each other to disturb the normal implantation and development of the embryo, thus causing stillbirth [26]. Long-term inflammatory stimulation in patients with endometriosis interferes with the normal contraction frequency and amplitude of the uterus, and endometriosis causes pelvic adhesions, leading to placenta previa [27]. Endometriosis pelvic adhesions reduce the amplitude of contraction of the myometrium, compromise postpartum uterine contraction, and increase the risk of postpartum hemorrhage [28]. Endometrial structural and functional changes, progesterone resistance, local estrogen and oxidative stress responses, and variations in inflammatory mediators and apoptotic markers all raise the risk of early placental abruption [29]. Patients herein were diagnosed histologically with endometriosis, which reduced the risk of misclassification.

The article "Adverse Pregnancy Outcomes Associated with Endometriosis and Its Influencing Factors" was retracted in 2023. Reasons: signs of a paper mill; compromised peer review; unreliable results or conclusions.

Swedish national research encompassing over 1.4 million singleton births found that women with endometriosis had a greater risk of preterm delivery, preeclampsia, placental problems, and cesarean delivery, but no link between endometriosis and fetal growth limitation was found. According to an Italian study, women with endometriosis are twice as likely to have a preterm delivery. The current study's findings are consistent with the prior research that revealed a link between endometriosis and placenta previa [30]. However, it is worth noting that the interaction between adverse pregnancy outcomes, such as placenta previa, and hypertensive disorders in pregnancy increases the risk of cesarean delivery and fetal growth restriction and may compromise the accuracy of the association between endometriosis and adverse pregnancy outcomes [31]. Furthermore, there are differences in the statistical methods used in different studies and the sample size, which also affect the research conclusion.

The present study is a single-center retrospective study, lacking a multicenter large sample control, and there are limitations in the representation of the association between endometriosis and pregnancy outcome, and further prospective multicenter cohort studies are needed to investigate the impact of endometriosis on maternal and infant outcomes. This study lacks analyses of the long-term effects on neonates. In future studies, the long-term follow-up of neonates is needed to more comprehensively describe the effects of endometriosis on neonatal outcomes. The present study lacks the study of the molecular mechanisms associated with endometriosis and adverse pregnancy outcomes, and the interaction mechanisms between the two will be further elucidated at the molecular level.

## 5. Conclusion

Endometriosis is an influential factor in adverse pregnancy outcomes and results in a high risk of preterm delivery, placenta previa, and cesarean delivery in patients. Mutual interactions exist among adverse pregnancy outcomes and thus require vigilance and appropriate management.

## Figures and Tables

**Table 1:** Patient characteristics ($\bar{x}$ ± *s*).

Groups	*n*	Ages (years)		Gravidity		BMI (kg/m^2^)		
		Scope	Average	Scope	Average	<18.5	18.5–23.9	>24
Study group	188	25–38	30.96 ± 3.32	1–3	1.56 ± 0.23	25	128	35
Control group	188	23–38	30.23 ± 2.98	1–3	1.41 ± 0.35	26	125	37
*t* value	—	—		—		—	—	—
*P* value	—	—		—		—	—	—

**Table 2:** Maternal pregnancy outcomes in both groups.

	Study group (*n* = 188)	Control group (*n* = 188)	OR (95% CI)	*P* value
Abortion	25	26	0.93 (0.58–1.44)	0.715
Ectopic pregnancy	1	2	0.69 (0.15–3.08)	0.651
Termination of pregnancy	1	1	0.68 (0.19–2.53)	0.541
Fetal death	2	1	6.32 (0.65–59.98)	0.121
Successful delivery	159	158	1.13 (0.73–1.74)	0.523

**Table 3:** Adverse pregnancy outcomes.

	Study group (*n* = 188)	Control group (*n* = 188)	OR (95% CI)	*P* value
Cesarean delivery	132	82	1.92 (1.33–2.85)	<0.001
Premature birth	18	5	2.43 (1.05–5.58)	0.029
Hypertensive disorder in pregnancy	10	11	0.77 (0.32–2.01)	0.611
Gestational diabetes	7	8	0.81 (0.41–1.99)	0.581
Anterior placenta	12	2	4.51 (1.23–16.50)	0.021
Premature abruption of the placenta	1	2	0.97 (0.70–1.33)	0.428
Fetal growth restriction	3	2	1.53 (0.21–9.98)	0.614
Luteal support	27	24	1.28 (0.72–2.24)	0.411

The article "Adverse Pregnancy Outcomes Associated with Endometriosis and Its Influencing Factors" was retracted in 2023. Reasons: signs of a paper mill; compromised peer review; unreliable results or conclusions.

## Data Availability

No data were used to support this study.
